The article "A Novel Evaluation Method of Static Balance Ability Based on Human Pelvic Center Measurement" was published in 2021. Journal: J Healthc Eng.

# A Novel Evaluation Method of Static Balance Ability Based on Human Pelvic Center Measurement

**DOI:** 10.1155/2021/6637963

**Published:** 2021-09-17

**Authors:** Mingli Xia, Shuai Guo

**Affiliations:** Department of Mechatronic Engineering and Automation, Shanghai University, Shanghai, China

## Abstract

This study evaluates the static balance ability of human body based on a lower limb rehabilitation robot. According to the balance parameters obtained from the movement trajectory of the center of human pelvis, SPSS statistical software was used to verify that there was a significant difference between the two groups (*p* < 0.01). Principal component analysis is used to allocate the weight of each parameter and establish the comprehensive evaluation value. The comprehensive evaluation value of the control group was 0.383 ± 0.038, and the experimental group was 0.875 ± 0.136. When the subject's comprehensive evaluation value is between 0.739 and 1.011, it indicates the presence of balance dysfunction, and when it is between 0.345 and 0.421, it indicates that the balance of the lower limbs of the subject is normal. Experimental results show that this evaluation method can objectively and quantitatively reflect the static equilibrium state of human body.

## 1. Introduction

It is of great significance to accurately assess the balance of patients with balance disorders in the clinical treatment of balance disorders and in the process of physician-assisted healthcare, so that different rehabilitation programs can be formulated to address the balance status, to ensure that the rehabilitation treatment is conducted simultaneously with the evaluation of the patients' rehabilitation effects, and to promote recovery for people with balance disorders [1].

The following methods are used to assess the body's balance ability: medical observation, scale assessment, and instrumental measurement [2]. Among them, the medical observation method is that the doctor observes the patient's balance performance under different conditions to assess directly. The advantage of this method is that it is simple to use and can be used to crudely screen patients without the use of equipment, but it is too subjective and the results are uncertain, and it does not quantify the criteria. The scale assessment method is to assess through a number of balance scales, such as the Berg Balance Scale, Tinetti Gait and Peace Scale, Fugl–Meyer Balance Function Scale, and Brunel Balance Scale. The advantage of this method is that it is simple to use and can be used to crudely screen patients without the use of equipment [3, 4], requires no instrumentation, and takes less time; the disadvantage is that it is prone to ceiling effects, and each option has blurred boundaries, making the results susceptible to subjective judgments, thus affecting the accuracy of the patient's balance assessment. Instrumental measurement is that with the development of computer technology, sensor technology, and electronic technology, quantitative measuring instruments are used in the assessment of balance ability. Terekhov, in 1976, first began to use pressure sensors to collect the human body pressure center COP position for balance ability analysis [5]. Nowadays, some scholars such as Sangeetha use the COP track extracted from the Nintendo Wii balance board [6] to evaluate the human body static balance and compare it with the Berg scale, and the results show that the balance ability results are consistent; there are also a number of scholars using the Technobody PK balance test and training system, such as the scholars Ren [7] and Song [8] based on the pressure sensor, to design a balance training instrument to analyze the human balance ability index and establish the balance scoring standard.

The article "A Novel Evaluation Method of Static Balance Ability Based on Human Pelvic Center Measurement" was published in 2021. Journal: J Healthc Eng.

From the analysis of the above contents, we know that most scholars currently use pressure sensors to obtain the center of pressure and extract pressure center-related parameters [9, 10]. The advantage of the pressure sensor is that it can accurately obtain the position and trajectory of the human body pressure center, but it lacks the balance parameters of the human body coronal plane. Therefore, this study adopts the maximum tilt angle as the balance parameter of the coronal plane for the first time. In order to evaluate the static balance ability of the human body accurately and effectively, this study uses the robot iReGo [11], designed by the research team to obtain the position changes of the human pelvic center and calculates the balance parameters by the balance algorithm.

## 2. Materials and Methods

### 2.1. System Design

The most important part of experimental equipment used in this study is the iReGo pelvic weight loss mechanism. The weight loss value of the pelvic weight loss mechanism can be set in order to reduce the burden of patients during training. However, the weight loss value was 0 when the experiment was conducted in this study. The pelvic weight reduction mechanism of the rehabilitation robot iReGo is shown in Figure 1. The force sensor and potentiometer obtain the displacement and angle change data of the robot in *x*, *y*, and *z* directions corresponding to the human body transverse plane, sagittal plane, and coronal plane, respectively.

By processing the output signal of the sensor, the real-time position of the pelvic center can be obtained. The pelvic center point is (*X*, *Y*), the initial pelvic center point is (*X*_0_, *Y*_0_), and the tilt angle is *θ*.

The article "A Novel Evaluation Method of Static Balance Ability Based on Human Pelvic Center Measurement" was published in 2021. Journal: J Healthc Eng.

Displacement variation of *Y*-direction:

(1) $$\begin{array}{c} Y=\frac{2\left(F1+F2\right)}{K}, \end{array}$$

where *F*1 is the output data of the left force sensor of the pelvic weight reduction mechanism, *F*2 is the output data of the right force sensor of the pelvic weight reduction mechanism, *K* is the spring beside the sensor of the pelvic weight loss mechanism, and the two sensors use the same stiffness linear spring.

Displacement variation of *X*-direction:

(2) $$\begin{array}{c} X=l\;\sin\left(\theta \right), \end{array}$$

where *θ* is the output data of the left and right potentiometer, and *l* is the length of the fixed short side of the pelvic four-bar mechanism.

Angle change of *Z*-direction:

(3) $$\begin{array}{c} Z_{\theta }=\theta , \end{array}$$

where *θ* is the output data for the upper and lower potentiometer.

### 2.2. System Verification

In order to verify the validity of the parameters obtained by the sensors on the pelvic weight reduction mechanism of the rehabilitation robot iReGo, the motion capture system is used as a reference, and synchronous experiments are used for verification and analysis. The experiment adopted a control experiment. The rehabilitation robot iReGo was placed in the field of view of the motion capture system. The subjects first wore the waist belt on the iReGo rehabilitation robot and then put the rigid body that can be recognized by the camera on the outer sides of the left and right waists. At the initial moment, the position of the waist on both sides and the corresponding were measured. For the position of the rigid body, the real-time position of the waist on both sides could be translated according to the rigid body data, and the motion capture mechanism calculated the center of travel position according to the positional relationship between the two rigid bodies. Within 30 seconds, the motion capture system and the rehabilitation robot iReGo collected data at the same time, as shown in Figure 2. By comparing the correlation and difference between the two sets of data, it is verified whether the data obtained by the sensor on the pelvic mechanism of the rehabilitation robot iReGo are valid.

### 2.3. Experimental Program

The subjects in the experimental group were patients with lower extremity balance dysfunction: 18 males, aged (50 ± 5) years, weighing 70 ± 10 kg, and height 170 ± 8 cm; and 12 females, aged 50 ± 5 years, weighing 55 ± 10 kg, and height 160 ± 6 cm. The subjects in the control group were healthy persons with lower limb function similar to the case group in gender, age, height, and weight.

The article "A Novel Evaluation Method of Static Balance Ability Based on Human Pelvic Center Measurement" was published in 2021. Journal: J Healthc Eng.

The person who wore the iReGo belt successfully, hung his/her hands naturally, stood with his feet 60° apart, and looked forward with both eyes. During the experiment, they were not allowed to talk with people or to be disturbed by external factors; otherwise, the experiment would be restarted.

As shown in Figure 3, after the preparation work was completed, click the start button on the iReGo balance system software on the screen to start the software and start collecting real-time centroid trajectory data. The iReGo balance system software displayed the subject's pelvic center position in real time as shown in Figure 4. The experiment time was 30 s. After the collection, the experimenter untied the belt.

According to the analysis of the pelvic center trajectory, the following nine parameters are selected as the parameters for balance measurement.

(1) Average swing: the average distance between the center of the pelvis and the initial point of the center of the pelvis. This article divides the parameter average swing into *x* and *y* directions:
  (4) $$\begin{array}{c} S_{a,x}=\sum \sqrt{\frac{{\left(x_{i}-x_{0}\right)}^{2}}{n}},\\ S_{a,y}=\sum \sqrt{\frac{{\left(y_{i}-y_{0}\right)}^{2}}{n}}, \end{array}$$
where (*x*_*i*_, *y*_*i*_) is the center point of the pelvis, (*x*_0_, *y*_0_) is the initial point of the center of the pelvis, *n* is the number of points; *S*_*a*,*x*_ is the average swing of *x*-direction, and *S*_*a*,*y*_ is the average swing of *y*-direction.
(2) Maximum swing: the maximum distance between the center of the pelvis and the initial point of the center of the pelvis. This article divides the parameter maximum swing into *x* and *y* directions:
  (5) $$\begin{array}{c} S_{m\text{,}x}=\text{Max}\left(S_{x}\right)\\ =\text{Max }|x_{i}-x_{0}\mathrm{|,}\\ S_{m,y}=\text{Max}\left(S_{y}\right)\\ =\text{Max }|y_{i}-y_{0}\mathrm{|,} \end{array}$$
where *S*_*x*_ is the distance of *x*-direction between the center of the pelvis and the initial point of the center of the pelvis, *S*_*y*_ is the distance of *y*-direction between the center of the pelvis and the initial point of the center of the pelvis, *S*_*m*,*x*_ is the maximum swing of *x*-direction, and *S*_*m*,*y*_ is the maximum swing of *y*-direction.
(3) Track length: the length of the trajectory of the center of the pelvis, that is, the sum of the distances between the center points of the adjacent pelvis.
  (6) $$\begin{array}{c} L=\sum_{i=1}^{n}\sqrt{{\left(x_{i}-x_{i-1}\right)}^{2}+{\left(y_{i}-y_{i-1}\right)}^{2}}. \end{array}$$
(4) Envelope area: the area enclosed by all swing points in the center of the pelvis. Envelope area algorithm idea first sort the points in the point set (the set of points in the whole experiment process) product method to obtain any simple polygon convex hull and finally calculate the envelope area by the combined triangulation method [12].
  (7) T=xiyi+1−yixi+1+xi+1y−iyi+1xi+xiyi−yixi,
where *T* is the variable for the concave-convex point discrimination. *T* > 0, then (*x*_*i*+1_, *y*_*i*+1_) is a convex point, *T* < 0, then (*x*_*i*+1_, *y*_*i*+1_) is a concave point, and *T* = 0, regarded as a neutral point, delete it. Calculate the area; the combined triangulation method sums the *S* area to be the envelope area.
  (8) Si−2=12xiyi−1−yixi−1+xi−1y−iyi−1xi+xiyi−yixi,
where *S*_*i*−2_ is the area of a triangle.
  (9) $$\begin{array}{c} S=\sum S_{i-2}, \end{array}$$
where *S* is the envelope area.
(5) Average swing speed: the speed at which the center of the pelvis swings per unit time indicates the speed of the body swing. This article divides the parameter average swing speed into *x* and *y* directions:
  (10) $$\begin{array}{c} V_{a,x}=\sum \frac{\left(\sqrt{{\left(x_{i}-x_{0}\right)}^{2}}\right)}{T},\\ V_{a,y}=\sum \frac{\left(\sqrt{{\left(y_{i}-y_{0}\right)}^{2}}\right)}{T}, \end{array}$$
where *V*_*a*,*x*_ is the average swing speed of *x*-direction, *V*_*a*,*y*_ is the average swing speed of *y*-direction, and *T* is the experiment time.
(6) Maximum tilt angle: the maximum angle formed by the vertical line when the body is inclined.
  (11) $$\begin{array}{c} \theta =\text{MAX}\left(Z_{\theta }\right), \end{array}$$
where *Z*_*θ*_ is the output data of *z*-direction potentiometer.

The article "A Novel Evaluation Method of Static Balance Ability Based on Human Pelvic Center Measurement" was published in 2021. Journal: J Healthc Eng.

## 3. Results

### 3.1. System Verification Results

The *Z*-direction roll angle of the rehabilitation robot (human coronal plane) and the data collected by the motion capture system are at the same time; the correlation between the two is calculated by Matlab *R* = 99.98%, the difference *p*=0, the maximum error is 0.4°, and the data are highly correlated as shown in Figure 5(a). The data of the *X*-direction displacement of the rehabilitation robot and the data collected by the motion capture system are at the same time; the correlation between the two is calculated by Matlab *R* = 99.98%, the difference *p*=0, the maximum error is 3.8 mm, and the data are highly correlated as shown in Figure 5(b). The data of the *Y*-displacement (human sagittal plane) of the rehabilitation robot and the data collected by the motion capture system are at the same time, the correlation between the two is calculated by Matlab *R* = 98.57%, the difference *p*=0, the maximum error is 2.5 mm, and the data height related are shown in Figure 5(c). The comparison with the data obtained by the motion capture system proves that the parameters obtained by the iReGo pelvic sensor are highly reliable and effective.

The article "A Novel Evaluation Method of Static Balance Ability Based on Human Pelvic Center Measurement" was published in 2021. Journal: J Healthc Eng.

### 3.2. Statistical Analysis

Different instruments and different postures have different balance indicators used in the research. Not any balance parameter can fully express a person's static balance. At the same time, the more parameters, the more able to describe a person's balance. However, the more parameters, the greater the possibility of information redundancy and the more mixed information; thus, the calculation costs too much. Therefore, we need a method to express all the parameters with one value. First, analyze the difference of the above balance parameters between the control group and the test group and eliminate the parameters that are not useful for the balance evaluation. This study is now based on the SPSSAU platform using the independent sample *t*-test analysis method to compare the differences of each parameter between the control group and the case group.

The *t*-test analysis using SPSSAU platform has the following difference results, as given in Table 1.

It can be seen from the above table that the experimental group and the control group are used to study the difference of track length, envelope area, average swing *x*, average swing *y*, maximum swing *x*, maximum swing *y*, average swing speed *x*, average swing speed *y*, and maximum tilt angle. From the above table, we can see that the different groups of track length, envelope area, average swing *x*, average swing *y*, maximum swing *x*, maximum swing *y*, average swing speed *x*, average swing speed *y*, and maximum tilt angle are all significant (*p* < 0.05), which means these nine parameters can be used for principal component analysis.

### 3.3. Comprehensive Evaluation Value

There is a certain amount of mixed information between the above balance parameters. It is necessary to establish a comprehensive evaluation value to replace the original multiple parameters to evaluate the static balance ability of the human body and quantify the parameter results. In this study, the principal component analysis method was used for analysis on different balance parameters. Remove information redundant factors, refine into new factors according to the weight of each parameter, and establish a comprehensive evaluation value for the new factors linearly weighted as the evaluation index. Through the analysis of the difference in the previous section, we can see that the track length, envelope area, average swing *x*, average swing *y*, maximum swing *x*, maximum swing *y*, average swing speed *x*, average swing speed *y*, and maximum tilt angle all have obvious differences. Based on this, the principal component analysis method of SPSSAU is used to establish a comprehensive evaluation value to replace the above nine parameters to evaluate the body's static balance ability. Take the control group as an example, and organize the data in the table into a standard normalized matrix for principal component analysis.  Table 2 is the variance explanation rate table after principal component analysis of the control group.  Table 3 is the component score coefficient matrix, which is extracted the weight of each factor.

The article "A Novel Evaluation Method of Static Balance Ability Based on Human Pelvic Center Measurement" was published in 2021. Journal: J Healthc Eng.

It can be seen from the above table that the principal component analysis has extracted a total of three principal components, and the characteristic root values are all greater than one. The variance interpretation rates of these three principal components are 42.874%, 28.815%, and 13.244%, respectively, and the cumulative variance interpretation rate is 84.933%. Their corresponding weighted variance interpretation rate, that is, the weight is 42.874/84.933 = 50.48%, 28.815/84.933 = 33.93%, and 13.244/84.933 = 15.59%. According to the table component score 1 (C_1), component score 2 (C_2), and component score 3 (C_3), the calculation formulas are as follows.

(12) $$\begin{array}{c} \text{C}\_1=-0.107L+0.190S+0.204S_{a,x}+0.132S_{a,y}+0.186,\\ S_{m,x}+0.213S_{m,y}-0.239V_{a,x}+0.061V_{a,y}-0.111A,\\ \text{C}\_2=0.295L+0.225S-0.163S_{a,x}+0.277S_{a,y}-0.074,\\ S_{m,x}+0.01S_{m,y}-0.002V_{a,x}-0.339V_{a,y}-0.156A,\\ \text{C}\_3=-0.303L+0.063S-0.228S_{a,x}+0.248S_{a,y}-0.541,\\ S_{m,x}+0.418S_{m,y}-0.227V_{a,x}-0.292V_{a,y}-0.157A. \end{array}$$

Therefore, the calculation formula of comprehensive evaluation value is

(13) $$\begin{array}{c} F=0.505\text{C}\_1+0.339\text{C}\_2+0.156\text{C}\_3. \end{array}$$

Among them, the statistical value of comprehensive evaluation value of the control group was 0.383 ± 0.038 and that of the experimental group was 0.875 ± 0.136. The data showed that the comprehensive evaluation value of the control group was higher than that of the experimental group, reflecting that the balance function of the control group was stronger than that of the experimental group and the comprehensive evaluation value is lower. Moreover, the comprehensive evaluation value of the control group fluctuated slightly, indicating that the control group had a strong ability of posture control. The comprehensive evaluation value obtained from the experiment is consistent with the characteristics of human balance function, which reflects the strength of subjects' balance function.

## 4. Discussion

There are many ways to measure static balance ability. Most scholars use the plantar pressure sensor to detect plantar pressure distribution. After obtaining the position (*x*, *y*) of the pressure center through the sensor, the parameters related to the pressure center are calculated according to the change of the pressure center, so as to evaluate the judgment ability of human body. However, due to the limitation of the plantar pressure sensor, only the parameters of *X* and *Y* planes can be calculated. The extracted parameters include the length of center of gravity track, the length of unit area track, the average swing amplitude, and the distribution ratio of center of gravity. However, human static balance is a three-dimensional overall balance, so it is very necessary to evaluate the static balance ability of human body with coronal balance data. In this study, three sensors of the iReGo pelvic weight loss mechanism can measure the data of three planes of human body. In this study, the maximum tilt angle of human body on coronal plane is added as one of the balance parameters to improve the evaluation of balance ability.

The article "A Novel Evaluation Method of Static Balance Ability Based on Human Pelvic Center Measurement" was published in 2021. Journal: J Healthc Eng.

The selection of balance parameters is the basis of balance ability evaluation. In this study, trajectory length, envelope area, average swing amplitude (*X*-direction and *Y*-direction), average swing speed (*X*-direction and *Y*-direction), maximum swing amplitude (*X*-direction and *Y*-direction), maximum swing speed, and maximum tilt angle are selected as balance parameters. It can be seen from Table 2 that there are significant differences in all parameters between the control group and the case group (*p* < 0.05).

In this study, the maximum tilt angle is used as a parameter to evaluate balance dysfunction for the first time. It can be seen from Table 2 that the maximum tilt angle has a significant difference between the control group and the experimental group, so it is correct to use it as the evaluation index. The experimental results provide an objective basis for the future application of the index. This study attempts to use principal component analysis to calculate the comprehensive evaluation value. Compared with the statistical value of the comprehensive evaluation value of the experimental group and the control group, the score of the control group is higher, and the floating of the score is small, which indicates that the control group is stronger than the case group in the stability of the center of gravity, and there is no big swing. Therefore, it is reasonable to apply principal component analysis to the field of balance function evaluation. The comprehensive evaluation value obtained is consistent with the characteristics of human balance function, which can reflect the strength of subjects' balance function.

The article "A Novel Evaluation Method of Static Balance Ability Based on Human Pelvic Center Measurement" was published in 2021. Journal: J Healthc Eng.

The traditional pressure plate can directly access the pressure center of human body, which is more convenient. The advantage of the rehabilitation robot is that it can obtain the three-dimensional data of the pelvic center. The data in this study are verified by the motion capture system, which is effective and accurate. The only disadvantage is that every time the subjects need to wear waist equipment, which is more complicated than the pressure plate test process.

## 5. Conclusion

In this study, a method for evaluating human static balance ability based on the pelvic center is discussed. The trajectory length, envelop area, average swing amplitude (*X*-direction and *Y*-direction), average swing velocity (*X*-direction and *Y*-direction), maximum swing amplitude (*X*-direction and *Y*-direction), maximum swing velocity, and inclination angle were selected as the evaluation parameters of the balancing ability. After analyzing the differences between the parameters of the control group and the experimental group, the principal component analysis method was used to fuse the selected evaluation parameters to obtain the independent principal component factors.

Finally, according to the variance contribution rate of each principal component factor, the weight of each principal component factor was determined, so as to obtain the comprehensive evaluation value of human static balance ability. By measuring and evaluating the balance function between the experimental group and the control group, the comprehensive evaluation value of the control group was 0.383 ± 0.038, and the comprehensive evaluation value of the experimental group was 0.875 ± 0.136. Results show that the center of the pelvic static balance evaluation method can evaluate the objective to evaluate the human body static balance ability, comprehensive evaluation value when the subject is within the scope of the experimental group (0.739, 1.011), the balance dysfunction, participants are required to further balance the rehabilitation training, within the scope of the control group (0.345, 0.421), show that the subjects lower limb equilibrium state is normal. This method has good clinical application potential in detecting patients' balance dysfunction, clarifying patients' balance recovery of lower limbs, and preventing falls. This study effectively solves the problem that the observation method and scale evaluation method cannot be used for quantitative analysis.

However, there are still a lot of further research works: first, to study the effects of visual and vestibular sensation related to human static balance; second, to find more objective and effective evaluation indicators, so that the detection of balance dysfunction can be more scientific and effective, and the balance ability can be assessed more correctly. Finally, expand the sample size to make the comprehensive evaluation value range of the control group and the case group more effective and accurate and promote the establishment of its evaluation criteria, so as to make the evaluation of static balance function more scientific and effective.

The article "A Novel Evaluation Method of Static Balance Ability Based on Human Pelvic Center Measurement" was published in 2021. Journal: J Healthc Eng.

## Figures and Tables

**Figure 1:** Pelvic weight loss mechanism.

**Figure 2:** Motion capture system verification.

**Figure 3:** Static balance ability measurement experiment.

**Figure 4:** Balance system software interface.

**Figure 5:** (a) The difference of *Z*-direction. (b) The difference of *X*-direction. (c) The difference of *Y*-direction.

**Table 1:** Balance parameter data of the control group and the test group.

	Test group	Control group	*t*	*P*
*L*	320.16 ± 30.06	243.31 ± 20.32	6.697	0.000^*∗∗*^
*S*	2.18 ± 0.36	0.79 ± 0.69	5.645	0.000^*∗∗*^
*S*_*a*,*x*_	0.04 ± 0.01	0.02 ± 0.01	3.628	0.002^*∗∗*^
*S*_*a*,*y*_	0.05 ± 0.00	0.02 ± 0.01	13.465	0.000^*∗∗*^
*S*_*m*,*x*_	0.36 ± 0.09	0.21 ± 0.05	5.109	0.000^*∗∗*^
*S*_*m*,*y*_	2.94 ± 1.03	0.96 ± 1.14	4.082	0.001^*∗∗*^
*V*_*a*,*x*_	3.16 ± 0.61	2.31 ± 0.20	4.179	0.002^*∗∗*^
*V*_*a*,*y*_	3.84 ± 0.42	1.27 ± 0.21	17.318	0.000^*∗∗*^
*θ*	2.03 ± 0.40	0.87 ± 0.25	7.689	0.000^*∗∗*^

^*∗∗*^ means that there is a significant difference between the control group and the test group.

**Table 2:** The control group variance explanation rate table.

No.	*λ*	Variance explained rate	Accumulation	*λ*	Variance explained rate	Accumulation
1	3.859	42.874	42.874	3.859	42.874	42.874
2	2.593	28.815	71.689	2.593	28.815	71.689
3	1.192	13.244	84.933	1.192	13.244	84.933
4	0.854	9.490	94.423	—	—	—
5	0.219	2.435	96.858	—	—	—
6	0.146	1.627	98.486	—	—	—
7	0.098	1.089	99.575	—	—	—
8	0.036	0.405	99.980	—	—	—
9	0.002	0.020	100.000	—	—	—

**Table 3:** Score coefficient matrix table.

Name	Component 1	Component 2	Component 3
*L*	−0.107	0.295	−0.303
*S*	0.190	0.225	0.063
*S*_*a*,*x*_	0.204	−0.163	−0.228
*S*_*a*,*y*_	0.132	0.277	0.248
*S*_*m*,*x*_	0.186	−0.074	−0.541
*S*_*m*,*y*_	0.213	0.010	0.418
*V*_*a*,*x*_	−0.239	−0.002	0.227
*V*_*a*,*y*_	0.061	−0.339	0.292
*θ*	−0.111	−0.156	−0.157

## Data Availability

The simulation results used to support the findings of this study are available from the corresponding author upon request.
